# 3D Reconstruction Method based on Medical Image Feature Point Matching

**DOI:** 10.1155/2022/9052751

**Published:** 2022-08-12

**Authors:** Jing Han, Yankun Cao, Lina Xu, Wei Liang, Qiyu Bo, JianLei Wang, Chun Wang, Qiqi Kou, Zhi Liu, Deqiang Cheng

**Affiliations:** ^1^School of Information and Control Engineering, China University of Mining and Technology, Jiangsu 221116, China; ^2^School of Software, Shandong University, Jinan 250101, China; ^3^School of Computer Science and Technology, Shandong Jianzhu University, Jinan 250012, China; ^4^Qilu University of Technology, Jinan 250353, China; ^5^Qilu Hospital of Shandong University, Jinan 250012, China; ^6^Optical Advanced Research Center, Shandong University, Qingdao 266237, China; ^7^School of Computer Science and Technology, China University of Mining and Technology, Jiangsu 221116, China; ^8^School of Information Science and Engineering, Shandong University, Qingdao 266237, China

## Abstract

Medical 3D image reconstruction is an important image processing step in medical image analysis. How to speed up the speed while improving the accuracy in 3D reconstruction is an important issue. To solve this problem, this paper proposes a 3D reconstruction method based on image feature point matching. By improving SIFT, the initial matching of feature points is realized by using the neighborhood voting method, and then the initial matching points are optimized by the improved RANSAC algorithm, and a new SFM reconstruction method is obtained. The experimental results show that the feature matching rate of this algorithm on Fountain data is 95.42% and the matching speed is 4.751 s. It can be seen that this algorithm can shorten the reconstruction time and obtain sparse point clouds with more reasonable distribution and better reconstruction effect.

## 1. Introduction

3D reconstruction is the core research part in the field of computer vision research. It is also an important part of medical image analysis. It uses the devices such as a camera to collect the image data of real scenes or hospital scanners to obtain medical image; uses the computer to automatically calculate and construct 3D geometrical model; and regains the 3D space information from 2D image information. It is widely applied to virtual reality [1], intelligent driving [2], smart home [3], medical treatment [4], preservation of cultural relics [5], etc. The research of related technologies is of great significance for intelligent diagnosis in medical images and HD 3D reconstruction of intraoperative navigation.

In medical image 3D construction, the method based on the structure from motion (SFM) has become the frequently used method of medical image 3D reconstruction and main research object in recent years. It is because of its convenience and the characteristic of having lower requirements for operation devices. The core idea of this method is extracting feature points from medical image for matching to restore the 3D information of image. Medical image matching is an important step of the 3D reconstruction method based on image. The matching accuracy directly affects the quality of 3D reconstruction. The nature of medical image matching is searching for the corresponding features between two images under the same scene. The medical image matching method based on feature points is currently the mainstream method of medical image matching. The excellent feature point matching method still demonstrates good adaptability to medical image transformation under complicated scenes, such as affine transformation, fuzzy, rotating and scaling, illumination, and compression scenes. Over the last decades, many scholars at home and abroad have introduced various methods and technologies to satisfy the requirements of match with stronger robustness and higher accuracy. The Harris detector [6] is a widely used detector of angular points and edge features. It constructs a Harris matrix based on the neighboring derivative of each point. However, its matching effect is hard to satisfy the requirements when medical image scale changes. Lowe [7] developed the widely used SIFT descriptor to find the unique image features. It is not sensitive to image scale and rotation and maintains good robustness in the aspects of noise, changing 3D scene viewpoints, illumination variation, and some other changes in a certain range. Therefore, it has become the frequently used method in the image feature point matching methods in 3D reconstruction. However, its calculation amount is large, which cannot satisfy the requirement for real-time matching. PCA-SIFT [8] and SURF [9] improved the SIFT algorithm on this basis. PCA-SIFT optimized the descriptor and accelerated the matching. SURF used a group of box filters to perform real-time matching for integral images. The ASIFT [10] proposed by YAN KE showed good robustness for the image with great viewpoint changes, achieving rather good matching effect. In recent years, the binary descriptors, such as FSAT [11], BRIEF [12], and ORB [13], have been widely applied in industry and have reduced the operation time. Yan et al. [14] performed normalization on the original SIFT descriptors and proposed a kind of elliptical neighborhood descriptor with affine invariant. Li et al. divided feature point neighborhood into annulus, at the same time accumulated the gradient directions at local coordinate system, and proposed a new feature descriptor CLCGH [15].

At present, the applications of 3D reconstruction have become wider and wider. Meanwhile, the requirements for its matching accuracy and velocity are also higher and higher. Many scholars and experts at home and abroad have conducted in-depth studies in the direction of 3D reconstruction based on medical image feature point matching. However, they still need to further explore the matching method with better performance. Therefore, the study on 3D reconstruction method based on medical image feature point matching is still the focus of this paper. The contributions of the paper are summarized in the following three points.

In this paper, the traditional SIFT algorithm is improved to solve the high-dimensional and false point problems for SIFT.

In this paper, through median filtering of the image, on the basis of the original SIFT detection of extreme points, the gradient is calculated by the Sobel operator, the division of the feature area is changed, and the dimension of the feature descriptor is reduced.

The algorithm proposed in this paper can improve the performance of the algorithm while reducing the computation time.

## 2. Materials and Methods

### 2.1. Improved SIFT Algorithm Based on Concentric Circle Neighborhood

#### 2.1.1. Improved Gradient Calculation of Sobel Operator

The precondition of accurately matching feature points is that the generated feature descriptors have good peculiarity. It means that it has stronger separating capacity compared to other points, and the feature descriptor vectors in adjacent areas are similar, while the ones in different areas are different. The differences in the image's geometric transformation and textural features have influences on the robustness of SIFT feature descriptors. The key points extracted by SIFT and the accounted neighborhood gradient histogram determine the features of feature descriptors. At the stage of feature matching, dissimilar feature descriptors may lead to errors in match. In this paper, the traditional SIFT method of calculating gradient magnitude and directions is improved, with new gradient definitions given to each pixel. At the stage of key point detection, it also uses traditional SIFT algorithm to detect the specific location of each key point.

For the images after two preprocessing methods of image graying and median filter, the Sobel operator [16], the discrete differential operator in essence, is adopted to calculate the gradient. Sobel operator combines Gaussian smoothing and differential derivative, which can effectively suppress noise, and is slightly influenced by image change. Besides, due to the simple calculation, it becomes the frequently used operator in edge detection and one of the approximate gradient functions based on image intensity. The DoG operator of SIFT algorithm has strong edge response, and the generated feature points contain many unstable edge response points. However, Sobel is one of the best edge detection operators. Therefore, Sobel operator is adopted to eliminate edge response to increase the anti-noise property of SIFT feature point. Firstly, it uses Sobel operator to define the image's gradient magnitude *G*_*σ*_^1^ in the Gaussian scale space:

(1) $$\begin{array}{c} G_{\sigma }^{1}=\sqrt{{\left(G_{x,\sigma }^{1}\right)}^{2}+{\left(G_{y,\sigma }^{1}\right)}^{2}}, \end{array}$$

where *G*_*x*,*σ*_^1^ and *G*_*y*,*σ*_^1^ represent the derivatives at horizontal direction *x* and vertical direction *y*, respectively, on the condition with the image scale factor of *σ*.

Next, the gradient size and direction of new feature points can be further obtained through the equation above:

(2) $$\begin{array}{c} G_{\sigma }^{2}=\sqrt{{\left(G_{x,\sigma }^{2}\right)}^{2}+{\left(G_{y,\sigma }^{2}\right)}^{2}}, \end{array}$$

(3) $$\begin{array}{c} G_{\sigma }^{2}=\arctan\left(\frac{G_{x,\sigma }^{2}}{G_{y,\sigma }^{2}}\right), \end{array}$$

where *G*_*x*,*σ*_^2^ and *G*_*y*,*σ*_^2^ are the derivatives of *G*_*σ*_^1^ at horizontal and vertical directions. Sobel operator calculates the horizontal derivative and vertical derivative of the equation above through conducting convolution operation on the image and templates at two directions. At the same time, it detects the image's vertical edge and horizontal edge information. The two templates are defined as

(4) $$\begin{array}{c} B_{x}=\left[\begin{array}{ccc} -1 & 0 & 1\\ -2 & 0 & 2\\ -1 & 0 & 1 \end{array}\right],B_{y}=\left[\begin{array}{ccc} -1 & -2 & -1\\ 0 & 0 & 0\\ 1 & 2 & 1 \end{array}\right]. \end{array}$$

#### 2.1.2. Feature Descriptor Based on Concentric Circle Neighborhood

The generation of feature descriptor in SIFT is the most time-consuming stage, so to reduce the complexity of operation, in this paper, the square neighborhood of 16∗16 of original SIFT is re-divided on the condition of not changing the size. Then, the square area with descriptors generated is replaced by a circle area, which is divided into eight subareas.

The feature points extracted by SIFT are the extreme values detected in Gaussian scale space, and the descriptors are generated in its neighborhood, which are the collection of local image information. Therefore, the more unique the descriptors, the richer the local image information, and the easier it is to realize image matching. The weight of pixel point in the neighborhood of feature point is related to its distance. The closer the pixel point is to feature point, the larger effect the feature point will have on it. Otherwise, the longer the distance, the smaller the effect. Therefore, a new neighborhood structure is proposed in this paper, which replaces the original square grid with eight concentric circle structure. Because the distance between the pixel point and feature point in the circular area is different, different weights are distributed to the pixel point. The main steps are as follows:

Step 1. The 16∗16 square neighborhood generated by original SIFT is replaced by 8-pixel circle structure. Sampling is conducted in the neighborhood range centering on key points, and the levels and gradient directions of the neighborhood pixels of feature points are defined to determine the predominating direction and auxiliary direction

Step 2. Taking the main direction of coordinate axis as starting point, its neighborhood is divided into 8 affine concentric circles by the unit of a radius. Taking 8-pixel as the maximum radius of a circle, the direction of each pixel is accounted. In the concentric circle area, the pixels in eight circles are assigned with different weights according to the distances from feature points for processing them, respectively, in the later matching stage

Step 3. For the concentric circles with different radiuses, centering on the feature point, the gradient accumulation method is adopted to represent feature descriptor. For each concentric circle' 8 directions uniformly distributed from 0℃ to 360℃, the gradient accumulation values are calculated, respectively. Finally, in 8 concentric circles, feature vectors are generated, i.e., 64-dimension descriptor

Step 4. Normalization of unit is performed on the generated 64-dimension feature vectors, to reduce the effect of illumination.  Figure 1 presents the optimized generated feature descriptor of concentric circle neighborhood. From Equations (2) and (3), it can obtain the main direction and the feature point's gradient value in the process of descriptor generation. Compared with original SIFT 128-dimension descriptor, the simplified descriptor can more abundantly describe the detailed information of image texture. It also can further highlight the peculiarity of feature points. The dimensions of feature descriptor are reduced by 50%, which can effectively reduce the complexity of operation

#### 2.1.3. Initial Matching of Feature Point Based on Neighborhood Voting

Through the sections above, the corresponding features and their descriptors are extracted from images. Next, similar feature vectors need to be found among these images, to determine the corresponding matching items. For 3D reconstruction, it needs the images shot from different viewpoints to completely cover the scenes. To associate these images totally, the initial matching of feature point is an essential step. In general, SIFT mainly adopts the ratio of nearest neighbor to the next nearest neighbor (NNDR) to perform the initial matching of feature point. Regarding this method, it uses Euclidean distance as the standard of unilateral matching, and it is simple and easy to realize. However, in this method, it can only use reference medical image to carry out one-way search for the similar features in target images. Meanwhile, any feature point involves multiple directions, and the matching of repeat point may occur during the matching, thus increasing the matching time. Therefore, on this basis, the NNDR approach is further extended in this paper. A rough matching method based on neighborhood voting is proposed. New constrictions are redefined for the initial matching point pair, to determine the corresponding initial matching items.

As the distance between pixel point and feature point is different, the pixel points are assigned with different weights. On this basis, a rough matching method based on neighborhood voting is proposed in this paper. The rationale is that the possibility of correct matching points in its neighborhood taking correct matching point as center is larger than the one of the neighborhoods taking mismatching point as center. According to the weight of the pixel point within matching point neighborhood to this point, the matching points are accumulated at the two constraints of distance and local direction for judging whether the point pairs corresponding to the reference medical image and the medical image to be matched are within the two set constraint ranges. The matching points satisfying the conditions are regarded as correct matching points, and the points are preserved. Otherwise, they are regarded as mismatching points, and the points are removed. The rough matching method based on neighborhood voting includes the following steps:

Step 1. 64-dimension feature description vectors contained by reference images and pending matching images are accounted. Inner product is performed on these vectors and the corresponding arc-cosine values are calculated. For the rough matching point, pairs obtained by NNDR method are sorted according to their corresponding matching qualities

Step 2. The matching points within correct matching point neighborhood are accounted at local main direction and distance, respectively. Through groups of experiments, it is shown that when direction threshold *T*_*θ*_ = 0.3, and distance threshold *T*_*d*_ = 0.4 are satisfied, more matching points can be preserved

Step 3. The distance *d* and main direction included angle difference Δ*θ* of any two initial matching points *ij* in the same image are calculated, respectively, as follows:

(5) $$\begin{array}{c} d=\sqrt{{\left(x_{j}-x_{i}\right)}^{2}+{\left(y_{j-}y_{i}\right)}^{2}}, \end{array}$$

(6) $$\begin{array}{c} \Delta \theta =\theta_{j}-\theta_{i}, \end{array}$$

where (*x*_*i*_, *y*_*i*_) and (*x*_*j*_, *y*_*j*_) represent the coordinates of any two matching points in the same image, respectively, and *θ*_*i*_, *θ*_*j*_ represent the angle where its main direction is

Step 4. Perform normalization operation by row vector for the reference images and pending matching images according to the distance value and direction included angle difference obtained in Step 3. Then, solve the corresponding distance inner product *dot*1 and direction included angle value *dot*2 between each matching point pair of two images. For example, as for matching point pair (*x*_*m*_, *y*_*n*_) and(*x*_*i*_, *y*_*i*_), the following can be obtained:

(7) $$\begin{array}{c} dot1=dot\left(im1\left(x_{m},y_{m}\right),im2\left(x_{i},x_{i}\right)\right), \end{array}$$

(8) $$\begin{array}{c} dot2=dot\left(im1\left(\theta_{m}\right),im2\left(\theta \right)\right). \end{array}$$

Step 5. Judge if the distance inner product and direction difference value obtained in Step 4 are within the two experience thresholds obtained in Step 2. If two values are both smaller than reference thresholds, then the matching point is preserved; otherwise, the point is removed

#### 2.1.4. RANSAC Algorithm and Optimization

For the unmatched points in initial matching point pairs, RANSAC algorithm is usually used to perform filter optimization. The advantage of RANSAC is that it can estimate the parameters of model fitting data by method of iteration in a group of observed values that contain inner values and abnormal values. It can reduce the effect of outliers on model parameters, thus effectively removing the abnormal values. As the number of iterations of RANSAC calculating parameters has no upper limit value, the time cost is rather high. It is assumed that the upper limit value is set for the number of iterations, perhaps the final results obtained are not optimal, and even probably wrong results can be obtained [17]. Therefore, it needs to set different thresholds according to practical conditions.

In this paper, the traditional RANSAC algorithm is improved. The rough matching points obtained by neighborhood voting are sorted according to the distance. The last 20% of points of all matching pairs are regarded as unqualified points, and then deleted. Besides, the remote point pairs are removed. Afterwards, RANSAC algorithm is used only on the remaining points. This algorithm aims to improve the probability of correctly matched points and, through reducing the number of samples to shorten the iteration time, obtain a new method of eliminating mismatching points, which is applicable to 3D reconstruction. The specific steps of the improved RANSAC algorithm are below, as shown in Figure 2:

Step 1. Calculate the distances of *N* pairs of matching points based on neighborhood voting. Sort them by the order of distance, and delete the last 20% of all points

Step 2. Randomly select 4 pairs of matching points from (0.8∗*N*) point pairs. In addition, the 4 pairs of matching points satisfy that any three points are non-collinear. Calculate the transformation matrix

Step 3. Through transformation matrix, calculate the distance d (set as 2 in this paper) when the remaining (0.8∗*N* − 4) matching point pairs match with the original corresponding matching points. The points less than the threshold *T* are regarded as inner points; otherwise, they are deleted

Step 4. Calculate the number of inner points obtained in Step 3. Then, fit the transformation matrix once again

Step 5. Before the inner points do not change, acquire the ultimate inner point set, and calculate new transformation matrix *H*

Compared to traditional RANSAC algorithm, the improved algorithm makes changes to the selected matching points. The probability of selecting correct matching points is increasing accordingly, thus reducing the effect of matching points on the required matrix. Meanwhile, the number of iterations is greatly reduced. The efficiency of removing false matching points is improved. The accurate matching points are preserved, and the precision of transformation matrix is improved as well.

## 3. Results and Discussion

The reconstruction of two images is the base of SFM reconstruction. In combination with the feature point extraction and initial matching methods proposed in Section 3 and mismatching point removing method proposed in Section 4, a new SFM reconstruction process can be obtained, as shown in Figure 3, with specific steps as follows:

Step 1. Firstly, the input reference images and images to be matched are preprocessed. It means performing graying and median filter operations to restrain the noise in images and guarantee the stability of the following reconstruction process

Step 2. SIFT algorithm is adopted to detect the extreme points in two images. Besides, Sobel operator is used to calculate the gradient of images. Then, the 64-dimension feature descriptor is generated based on concentric circles neighborhood; the feature vector and location information of feature points of the two images are saved

Step 3. Neighborhood voting method is adopted to carry out initial matching of feature points for the two images. In addition, the initial matching point set of all features is saved

Step 4. The improved RANSAC algorithm is used to optimize the initial matching point set and to remove the dismatching points contained, obtaining the ultimate matching point set

Step 5. The basis matrix *F* is solved based on RANSAC eight-point method. In combination with camera internal reference *K*, the transformation relation *E* = *K*′^*T*^*FK* is used to obtain the basis matrix: Essence matrix [18]*E* with special form under the normalized medical image coordinate system. Then, perform SVD (singular value decomposition) [19] of *E* = *UDV*^*T*^ (*U*, *V* are both 3∗3 orthogonal matrix, *D* = diag(*r*, *s*, *t*) is diagonal matrix) on Essence matrix *E*. This aims to determine the moving posture of camera, i.e., rotation matrix *R* and translation vector *T*

Step 6. After several steps, the internal and external parameters of camera are obtained. *P*_1_ = *K*[1|0] and *P*_2_ = *K*[*R*|*T*] are used to determine each projection matrix of two images. Under the condition that the internal and external parameters of camera and accurate matching points locations are known, the Triangulation method can be used to further determine the corresponding spatial discrete 3D point coordinate *M* of matching point pairs *m* and *m*′ in the relation of projection matrix *P*_1_*M* = *m* and *P*_2_*M* = *m*. Finally, a new medical image is added to each group. The above steps are iterated through SFM until the 3D coordinates of matching points of three images are obtained, thus realizing the 3D reconstruction of images.

Figures 4 and 5 are Fountain image and David head image which is usually used in 3D reconstruction, which are from the database of Swiss Federal Institute of Technology. Experiments are carried out on the images by using the method of this paper and Literature [20], respectively, to verify the advantages of this method proposed in this paper.  Figure 6 is the image of different slices of cardiac ultrasound. It can be seen from the figure that different sections of medical images and natural images from different angles have something in common. In natural images, three-dimensional reconstruction can be performed by means of feature matching, and the same principle can be applied to medical images.

### 3.1. Feature Point Extraction and Initial Matching Experiments

Firstly, preprocessing is performed on Figures 4 and 5. Then, SIFT algorithm is used to detect the extreme points, and Sobel operator is used to calculate the gradient of images. At the same time, through the feature vectors generated by concentric circles neighborhood, the initial matching is carried out based on neighborhood voting method. The initial matching results are obtained, as shown in Figure 7.

It can be shown from Figure 6 and Table 1 that the initial matching performance by this method is generally better than that by Literature [20] method. In terms of correct matching rate, this method can reach above 94%, while Literature [20] method is obviously lower. Regarding matching time, this method has shorter elapsed time. The number of matching points extracted in this paper is superior to that by the SIFT algorithm adopted in Literature [20] method, and the distribution is more uniform, and stable matching point pairs are obtained. Meanwhile, it shows many obvious slashes from the initial matching images of Literature [20], which are the point pairs generated by mismatching. SIFT algorithm is adopted to complete the extraction of feature points, and at the same time, the nearest neighbor search algorithm based on Euclidean distance and feature vector included angle [21] is used to perform initial feature point matching. The obtained matching points are not uniformly distributed, and it is hard to find correct initial matching point pairs. Moreover, high-dimension descriptors make the matching efficiency low. Hence, the matching effect is unsatisfactory. In this paper, the neighborhood region shape of descriptors is changed; the original square grid is replaced by eight concentric circles structure; the 128-dimension descriptor of SIFT is reduced to 64 dimensions; two constraints, i.e., distance and direction, are used to optimize the initial matching point pairs. Compared with the nearest neighbor search method proposed in Literature [20], more matching points are searched, thus improving the matching efficiency and showing an obvious matching advantage. Therefore, it can be seen from experimental results and image initial matching effects that this method has better initial matching effect than Literature [20] method. While it obtains high matching accuracy, the arithmetic speed is also improved correspondingly.

### 3.2. Experiments of Removing Mismatching Points

In this section, the initial matching results in the last section are optimized, i.e., the experiments of removing mismatching points are carried out. It aims to preserve stable and accurate matching point pairs, thus utilizing the consequent 3D reconstruction.  Figure 8 is the experimental results of mismatching point removing by this method and Literature [20] method.

Through observing the accurate matching effect, it can be known that the traditional RANSAC algorithm was adopted in Literature [20], and this method can both remove the repeated and large error points in the initial matching points. As the reference images and images to be matched obtained by the former one still have a certain quantity of mismatching point pairs, the two images have elapsed time of 9.193 s and 8.380 s, respectively. The feature point optimization method proposed in this paper can remove more mismatching points and preserve more accurate matching points, with elapsed time of 7.589 s and 7.132, respectively. The arithmetic speed is improved as well. RANSAC uses the principle of iterations for all initial matching point pairs to remove the unqualified interference matching points. Therefore, when there are plenty of repeated point pairs in images, the whole computation time of RANSAC will also increase. By contrast, the method in this paper has good adaptation to this condition. It can satisfactorily accomplish the task of removing mismatching points. Therefore, it is easier to further obtain the 3D reconstruction effect with higher accuracy. To sum up, the method in this paper guarantees the validity and stability of accurate matching, further enhancing the stability of consequent 3D reconstruction.

### 3.3. 3D Sparse Reconstruction Experiment

Based on the above image feature point extraction and matching experiments, next, an image is added to each group. SFM iteration is used to carry out 3D sparse reconstruction experiment. The 3D sparse point cloud results obtained by the reconstruction of the above targets are shown in Figures 4–6.

Literature [20] uses SIFT algorithm to search for the feature points in images. Then, the least square method is adopted to obtain the coordinates of 3D space. It can be seen from above figures that the final amount of point cloud obtained by Literature [20] method is smaller than that by this method. In terms of reconstruction effect, this method can basically restore the main profile of images. Meanwhile, the processing effect of some image details is better. Especially, the part of David head in Figure 9 obviously has fewer noisy points, while Literature [20] method causes the loss of more detailed information, and the obvious cavitation will occur. For example, for the reconstruction part of Fountain, the reconstruction effect is not satisfactory. It is because in this paper, on the basis of image preprocessing, Sobel operator evades the noise as well, reducing the effect of noise on reconstruction. The improved SIFT extracts more feature points. The improved initial matching and mismatching point removing method better optimize matching points. Therefore, the quality of point cloud is relatively high. Regarding the elapsed time of reconstruction, the time of reconstruction image by this method is 39 s and 27 s, respectively, while that with the other method is 50s and 34 s, respectively. This method reduces half of the dimensions for descriptors, which is superior to the other method in reconstruction efficiency. Hence, it is better than the reconstruction method in Literature [20] both in the whole reduction degree and accurate descriptions of details. It can obtain the sparse point cloud with more reasonable distribution and better reconstruction effect. In addition, the time is correspondingly shortened. In general, satisfactory effects have been achieved in the reconstruction result in this paper. Due to the excellent performance of this feature point matching, this method can be completely applied to medical images, which has solved the problem of three-dimensional reconstruction of medical images.

## 4. Conclusions

In this paper, it proposes an improved SIFT matching 3D medical reconstruction method. It carried out studies on the aspects of improving the image feature point extraction and initial matching performance in 3D reconstruction, and the aspect of removal methods of optimizing mismatching points as well. Firstly, SIFT algorithm is adopted to detect the specific location of each key point. Meanwhile, Sobel operator is used to calculate the gradient of computer images, replace the original square grid with eight concentric circles structure, and generate 64-dimension descriptor based on concentric circle neighborhood. Secondly, it proposes an initial matching method of feature point based on neighborhood voting in terms of initial matching strategy. It uses simplified RANSAC algorithm to regard the last 20% of all initial matching point pairs obtained through neighborhood voting as unqualified points, which are deleted. Eventually, it realizes the 3D sparse reconstruction of image and obtains the sparse point cloud with more reasonable distribution and better reconstruction effect. Experimental results indicate that this method can obtain sparse point cloud with more reasonable distribution and better reconstruction effect, and the time is also correspondingly shortened. Generally speaking, this paper has achieved satisfactory effects in the reconstruction results. Moreover, it is verified that the image matching method proposed in this paper has the feasibility and effectiveness to the medical image reconstruction results.

## Figures and Tables

**Figure 1:** Improved SIFT feature descriptors.

**Figure 2:** Flow chart of improved RANSAC algorithm.

**Figure 3:** Basic process of 3D reconstruction based on image.

**Figure 4:** Fountain image.

**Figure 5:** The David head image.

**Figure 6:** Schematic diagram of different slices of cardiac ultrasound.

**Figure 7:** Feature point extraction and initial matching experiment results.

**Figure 8:** Experimental results of mismatching point removal.

**Figure 9:** Reconstruction results.

**Table 1:** Feature point extraction and initial matching experiment results.

Experiment image	Matching method	Initial matching rate/%	Initial matching time/s
Fountain	Literature [20]	90.56	6.521
	This method	95.42	4.751
David	Literature [20]	82.78	6.334
	This method	94.89	4.174

## Data Availability

The data used to support the findings of this study are currently under embargo, while the research findings are commercialized. Requests for data, 12 months after publication of this article, will be considered by the corresponding author.
